RETRACTED

# Efficacy Investigation of TACE Combined with Lenvatinib and Sintilimab in Intermediate-Stage Hepatocellular Carcinoma

**DOI:** 10.1155/2022/6957580

**Published:** 2022-07-06

**Authors:** Menglong Zhang, Weiguo Lai, Jian Zhang, Bijuan Hu, Liyin Huang, Cunkun Chu

**Affiliations:** ^1^Ganzhou People's Hospital, No. 16, MeiGuan Road, Zhanggong District, Ganzhou, 341000 Jiangxi, China; ^2^Library, Shandong First Medical University & Shandong Academy of Medical Sciences, Tai'an, 271000 Shandong Province, China

## Abstract

**Objective:**

To evaluate the effectiveness of transarterial chemoembolization (TACE) combined with lenvatinib and sintilimab in treating patients with midstage hepatocellular carcinoma (HCC).

**Methods:**

Sixty-two patients with midstage HCC were enrolled in this study. All of them were firstly treated in our hospital between September 1, 2019, and March 1, 2020. According to different treatment regimens, they were divided into the control group (31 cases, TACE group) and the observation group (31 cases, TACE combined with lenvatinib and sintilimab group). Each patient was followed up for at least 30 months to compare the short-term clinical efficacy and survival rate between the two groups.

**Results:**

The objective response rate (ORR) and disease control rate (DCR) of the observation group at 3 months were 77.4% and 93.5%, respectively, which were higher than those of the control group (*P* < 0.05). The 2-year cumulative overall survival rate of the observation group was 64.5%, which was significantly higher than that of the control group (*P* < 0.05). The survival curve of the disease-free survival rate in the observation group was higher than that in the control group, and the difference was statistically significant (*X*^2^ = 4.313, *P* < 0.05).

**Conclusion:**

TACE combined with lenvatinib and sintilimab in the treatment of Barcelona Clinic Liver Cancer (BCLC) stage B hepatocellular carcinoma can effectively control the tumor progression and prolong the survival time of patients. Those preliminary findings need validation in larger studies, with a prospective design and longer follow-up.

## 1. Introduction

Hepatocellular carcinoma (HCC) is the sixth most commonly diagnosed and fourth most lethal neoplasm worldwide. The incidence of HCC has doubled over the past two decades, especially in the United States, Europe, Japan, and China [1]. According to the Barcelona Clinic Liver Cancer (BCLC) staging standard, HCC is divided into four stages, of which stage B is equivalent to the intermediate stage of Tumor Node Metastasis (TNM) staging. The treatment of patients in this stage is more complex than that in the early stage, and their prognosis is better than that in the advanced stage, so special attention should be paid to it.

RETRACTED

At present, both the European Association for the Study of the Liver (EASL) [2] and the American Association for the Study of Liver Diseases (AASLD) [3] recommend transarterial chemoembolization (TACE) as the standard treatment option for patients with intermediate-stage (BCLC stage B) HCC. However, TACE can induce hypoxia and increase the level of VEGF in HCC, which may be the driving factor of tumor growth, progression, and metastasis [4, 5]. Molecular targeted drugs, as multikinase inhibitors, may inhibit tumor angiogenesis and tumor cell proliferation [6], among which lenvatinib proved to prolong the progression-free survival (PFS) of patients with intermediate-stage HCC refractory to TACE [7] and was approved for first-line treatment of unresectable hepatocellular carcinoma (uHCC) based on the REFLECT study [8]. Meanwhile, sintilimab is a human immunoglobulin G4 (IgG4) monoclonal antibody that specifically binds to the programmed death-1 (PD-1) molecule on the surface of T-cells, consequently blocking the tumor immune tolerance-inducing PD-1/programmed death-ligand 1 (PD-L1) pathway, reactivating the antitumor activities of lymphocytes, and inhibiting tumors [9]. Application of anti-PD-1/PD-L1 antibodies as checkpoint inhibitors is rapidly becoming a promising therapeutic approach in treating tumors, and some of them have successfully been commercialized in the past few years [10].

Combination therapies have been researched for liver cancer, with synergistic effects [11], including PD-1 inhibitors plus lenvatinib and TACE plus lenvatinib [12, 13]. However, to date, TACE combined with lenvatinib plus sintilimab has not been studied for patients with BCLC B-stage HCC. Therefore, we conducted this retrospective study to assess the efficacy and safety of TACE combined with lenvatinib plus sintilimab in BCLC B-stage HCC. This preliminary study was aimed at evaluating the effectiveness of TACE combined with lenvatinib and sintilimab in treating patients with midstage HCC. It was hypothesized that the combination of TACE with lenvatinib and sintilimab would be superior against TACE alone.

## 2. Patients and Methods

### 2.1. Patients

In this retrospective study, sixty-two patients with HCC admitted to the Department of Minimally Invasive Interventions and the Department of Oncology of Ganzhou Hospital affiliated to Nanchang University between September 1, 2019, and March 01, 2020, were included. All patients were required to complete clinical information, and both patients and families cooperated with the follow-up. All patients were informed verbally and in writing on the study and provided their informed consent; this procedure and the whole study protocol has been reviewed and approved by the local ethics committee. Based on the Chinese Hepatocellular Carcinoma Diagnosis and Treatment Standard, all patients were diagnosed with HCC by histopathological or clinical diagnosis. The inclusion criteria for patients in this study were (1) aged between 18 and 75 years; (2) patients with pathologically histologically or clinically confirmed HCC; (3) BCLC staging B; (4) ECOG performance status less than 2; (5) Child-Pugh class A or B; no extrahepatic metastases and/or macrovascular invasion; (6) no prior TACE/Hepatic Artery Infusion Chemotherapy (HAIC) and I-125 particle implantation or systemic therapy (including systemic chemotherapy, molecular targeted therapy, immunotherapy with cytotoxic T lymphocyte-associated antigen-4 (CTLA-4), and PD-1/PD-L1); (7) intrahepatic reproducible lesions according to the modified Response Evaluation Criteria In Solid Tumors (mRECIST) [8]. The chronological order of the start of the three therapies of TACE, sintilimab, and lenvatinib is not required, but after the first therapy starts, the other two therapies must be completed within 1 month. Exclusion criteria were (1) portal vein trunk cancer thrombosis formation; (2) severe cardiac, pulmonary, and renal diseases, cachexia, or multiorgan failure; (3) expected survival time < 3 months; (4) gestation; (5) other tumors; (6) interrupted follow-up or missing information data; and (7) premature discontinuation of systemic therapy due to drug response (within 3 months).

RETRACTED

### 2.2. TACE

TACE was performed using the Seldinger technique, and a catheter was placed in the celiac artery or common hepatic artery for angiography. After acquiring images of the arterial phase, parenchymal phase, and venous phase, we can figure out the anatomical shape of hepatic artery, the presence or absence of vascular variation, and the location, size, quantity, blood supply type, and presence of arteriovenous fistula of then hepatic parenchyma tumor. Then, super selective cannulation to the tumor-feeding arteries for angiography was performed. Depending on the size of the tumor, the appropriate amount of chemotherapeutic drugs (20-40 mg of lobaplatin, 20-40 mg of epirubicin) was mixed with 10 ml of poppy lipiodol to embolize the tumor blood vessels. After the tumor vessel was saturated and the portal vein branches around the lesion were stagnant, 300-500 *μ*m PVA particles were slowly injected until the blood flow stopped, so as to achieve complete tumor embolization or staged compression embolization. Postoperative hepatoprotective support and symptomatic management were provided. The interval of TACE treatment was determined by imaging review.

RETRACTED

### 2.3. Lenvatinib

Patients received lenvatinib (Patheon Inc., H20180052) orally within one month after the first TACE, at a dose of 12 mg/d (weight ≥ 60 kg) or 8 mg/d (weight < 60 kg) until tumor progression, patient death, or intolerable adverse drug reactions. Adverse drug reactions include the following: increased blood pressure, gastrointestinal reactions, thyroid dysfunction, and albuminuria, which are graded according to NCI-CTCAE version 4.03 [14]. For grade 3 or 4 adverse events, we performed symptomatic treatment first, and if there was no improvement, then the dose of lenvatinib was reduced to 8 mg/d and 4 mg/d or 4 mg every other day. The treatment was interrupted if intolerable adverse events persisted.

### 2.4. Anti-PD-1 Inhibitors

Patients should receive the first injection of sintilimab (Innovent Biologics, Ltd., S20180016) within 1 week before discharge and then every 3 weeks thereafter. The dose and method of each administration is sintilimab 200 mg with 100 ml of saline and intravenous infusion for 30 minutes. Adverse drug reactions include macular papules, itchy skin, gastrointestinal reactions, hepatic impairment, thyroid dysfunction, rash, immune pneumonia, reactive capillary hyperplasia, and discontinuation of dosing if still intolerable after symptomatic treatment.

### 2.5. Follow-Up Visits

Follow-up visits were required after the TACE procedure. The patients were followed up by inpatient or outpatient during 1 month. The deadline for follow-up was March 1, 2022. The follow-up included physical, laboratory, and imaging examinations, as well as adverse reactions. Laboratory examinations included blood routine tests, blood biochemistry tests, alpha-fetoprotein (AFP), coagulation function tests, liver and kidney function tests, thyroid function tests, and other tests. Imaging examinations include enhanced MRI of the upper abdomen and chest CT. For patients with residual tumor or recurrence detected by imaging and AFP, follow-up interventional therapy was considered. The indications for re-TACE were as follows: Child-Pugh class A or B, ECOG score 0 or 1, prothrombin prolongation time < 4 s, and platelet count > 109/l.

### 2.6. Evaluations

The efficacy of cases was evaluated after each treatment and follow-up with reference to the mRECIST [15]. Complete response (CR) was defined as disappearance of all target lesions maintained for more than 4 weeks; partial response (PR) was defined as ≥30% reduction in the total diameter of target lesions maintained for more than 4 weeks; disease progression was defined as ≥20% increase in the total diameter of target lesions or the appearance of new lesions; and stable disease was defined as reduction not reaching partial remission or increase not reaching disease progression. The target lesion was defined as the selected arterial phase enhancement lesion on MRI. Based on this, the objective response rate (ORR), stable disease (SD), and disease control rate (DCR) were calculated, which were defined as ORR = (CR + PR)/total cases × 100% and DCR = (CR + PR + SD)/total cases × 100%. Progression-free survival (PFS) was defined as the time from the first treatment to diagnosis of disease progression or death or the end of follow-up; overall survival (OS) was defined as the time interval from the first treatment to death or the end of follow-up. Based on this, cumulative survival and cumulative progression-free survival were calculated.

RETRACTED

### 2.7. Statistical Analysis

The differences in the clinical characteristics between two groups were assessed by Student *t*-test and chi-square test. The Kaplan-Meier method was used for survival analysis to plot survival curves, and log-rank test was used for comparison of survival rates. *P* < 0.05 means the difference is statistically significant. All statistical analyses were performed with SPSS version 20.0.

## 3. Results

### 3.1. Basic Treatment

In total, 62 HCC patients were enrolled in this study, including 31 in the observation group and 31 in the control group. Each patient was followed up for 24 months. The comparison of baseline data between the two groups is shown in Table 1. There were no statistically significant differences in gender, age, weight, tumor-related characteristics (number and size), hepatitis B virus (HBV) infection, AFP levels, Child-Pugh class, and ECOG score between the two groups (*P* > 0.05). In the observation group, 4 patients stopped taking medicine due to drug reaction during the study period.

### 3.2. Short-Term Efficacy

All 62 patients completed interventional surgery successfully. One patient developed liver abscess 1 week after operation and 42 patients developed postembolization syndrome such as abdominal pain, fever, nausea, and vomiting, while the other patients did not have obvious complications.

According to mRECIST, CR, PR, SD, progressive disease (PD), ORR, DCR, and other efficacy indicators of patients in the observation group and the control group at 1 and 3 months after surgery were counted and compared (Table 2). The ORR and DCR of the observation group at 3 months were 77.4% and 93.5%, respectively, higher than those of the control group, and the difference between the two groups was statistically significant (*P* < 0.05).

### 3.3. Survival Analysis

All 62 patients completed 2-year follow-up and the follow-up span was 30 months. Disease progression occurred in 46 patients during follow-up (20 in the observation group and 26 in the control group). Thirty patients died (11 in the observation group and 19 in the control group), including 25 deaths due to tumor progression, 3 deaths due to liver failure, 1 death due to upper gastrointestinal bleeding, and 1 death due to cerebrovascular accident. The six-month, 1-year, and 2-year cumulative overall survival rates of the observation group are shown in Table 3 and Figure 1, which were equal to or higher than those of the control group. The difference in 2-year overall survival rate of the two groups was statistically significant (*P* < 0.05). The progression-free survival curves of the observation group and the control group are shown in Figure 2. It was obvious that PFS in the observation group was higher than that in the control group, and the difference between the two groups was statistically significant (*X*^2^ = 4.313, *P* < 0.05).

RETRACTED

## 4. Discussion

In this study, we investigated the feasibility and efficacy of TACE combined with lenvatinib and sintilimab in the treatment of intermediate-stage HCC. It was found that the one-year survival rate and two-year survival rate of patients treated with this regimen could reach 80.6% and 64.5%, respectively. This is a significant improvement compared with TACE alone. It can be a reliable option for HCC patients. This result is determined by the role of interventional therapy, molecular targeted therapy, and immunotherapy and can be deduced from the perspective of pathophysiology and pharmacology.

TACE is an effective treatment option for intermediate stage (BCLC B) HCC [16, 17]. However, repeated TACE may lead to liver function impairment and even TACE resistance [18, 19], and most patients have a poor prognosis [20]. According to the six-and-twelve model, BCLC stage B hepatocellular carcinoma with tumor load > 6 showed poor prognosis after TACE treatment [21]. For these patients, TACE combined with targeted therapy should be a promising option. TACE combined with lenvatinib had been used in HCC for a long time and showed improved effectiveness [22, 23]. The possible mechanism is that TACE induces angiogenesis and enhances the serum concentrations of vascular endothelial growth factor (VEGF) because of local hypoxia. Lenvatinib is an inhibitor for tyrosine kinase receptor (RTK), which can inhibit the kinase activity of VEGF receptors such as VEGFR1 (Flt1), VEGFR2 (KDR), and VEGFR3 (Flt4) [24]. In addition, it can also inhibit other RTKs related to angiogenesis and tumorigenesis pathways, including fibroblast growth factor (FGF) receptors, such as fibroblast growth factor receptor (FGFR)1, 2, 3, and 4, and platelet-derived growth factor (PDGF) receptors such as PDGFR-*α*, KIT, and RET [25, 26]. We can summarize that lenvatinib may exert its greatest antiangiogenic effects before or after TACE.

RETRACTED

PD-1 receptor expressed by T cells can inhibit T cell proliferation and cytokine production by binding to its ligands, PD-L1 and PD-L2. For some tumor cells, when PD-1 ligand is upregulated, the immune monitoring of activated T cells can be inhibited through this signal transduction pathway [27–29]. Sintilimab is a human IgG4 monoclonal antibody. It can bind to the PD-1 receptor, block the immunosuppressive response mediated by its interaction with PD-L1 and PD-L2, and enhance the antitumor immune effect. In the mouse tumor model, tumor growth can be inhibited by blocking the activity of the PD-1 pathway [30, 31]. Nowadays, the PD-L1 pathway blockade has become a promising and favorable immunotherapy for adjusting host immune responses and inhibiting the development of HCC [32, 33].

In this study we can find that short-term efficacy indexes such as ORR and DCR of the observation group in each period were higher than those of the control group. There was no significant difference between the two groups at 1 month (*P* > 0.05). With the extension of time, there was significant difference between the two groups at 3 months (*P* < 0.05). This result may be attributed to the respective pharmacological mechanism of TACE, lenvatinib, and sintilimab. TACE alleviated the disease mainly by blocking the blood supply of the tumor, and it played a key role in the early stage, so there was no significant difference in ORR and DCR between the two groups in 1 month. With the emergence of neovascularization and the recovery of tumor microenvironment, lenvatinib and sintilimab gradually took the lead in treatment [34, 35], so ORR and DCR in the observation group began to be significantly higher than those in the control group after 3 months.

There were several limitations in this study. Firstly, this was a retrospective trial with a limited sample size, which may lead to potential bias. In the absence of a sample size calculation, and according to the unclear robustness of the conclusions in this study, the findings must be seen as preliminary results. Secondly, the treatment options in this study were determined according to the preferences of doctors or patients, which may lead to the selection bias of our study population. Thirdly, follow-up period was relatively short and the outcome for some patients has not been obtained, so it was impossible to fully evaluate PFS and OS. Fourthly, in this study, the combination regimen was only compared with TACE alone. Next, we will conduct a multivariate analysis of the efficacy among TACE, lenvatinib, and sintilimab. In addition, there are some limitations regarding the inclusion and exclusion criteria. Thereby, patients with an age over 75 years were included to eliminate high age as a potential confounder. Overall, as mentioned above, this is a preliminary study, which requires further validation in larger studies with higher follow-up periods.

RETRACTED

## 5. Conclusion

Within the limitations of this preliminary study, the blood flow of the tumor can be blocked by TACE to the greatest extent. Lenvatinib can effectively inhibit neovascularization and reduce collateral circulation; at the same time, sintilimab can effectively activate T cells and enhance immune response. TACE combined with lenvatinib and sintilimab appears to be an effective method for the treatment of intermediate HCC.

## Figures and Tables

**Figure 1:** Kaplan-Meier estimates of overall survival (OS) by mRECIST.

**Figure 2:** Kaplan-Meier estimates of progression-free survival (PFS) by mRECIST.

**Table 1:** Baseline characteristics of the two groups.

	Observation group	Control group	*P*
Gender (male/female)	21/10	19/12	0.791
Age ($\bar{x}\pm s$)	58.8 ± 12.1	56.7 ± 10.6	0.721
Weight ($\bar{x}\pm s$)	62.5 ± 5.8	65.6 ± 6.9	0.188
Tumor number^∗^ (one/more)	20/11	24/7	0.402
Tumor diameter^∗∗^ (<5 cm/>5 cm)	9/23	12/19	0.430
History of hepatitis B (yes/none)	28/3	27/4	0.688
AFP (negative/positive)	5/28	4/27	0.612
Child-Pugh score (A/B)	18/13	20/11	0.795
Score of ECOG (0)	31	31	1.000

AFP: alpha-1-fetoproteine; ECOG: Eastern Cooperative Oncology Group. Note: ^∗^the number of tumors is the number of tumors that can be measured. ^∗∗^Tumor diameter is the sum of all target lesion diameters measured for each case based on measurements provided by mRECIST.

**Table 2:** Comparison of short-term treatment effects between the observation group and the control group.

Curative effect	1 month			3 months		
	Observation group	Control group	*P*	Observation group	Control group	*P*
CR	18 (58.1%)	19 (61.3%)		15 (48.4%)	10 (32.3%)	
PR	10 (32.3%)	7 (22.6%)		9 (29.0%)	6 (19.4%)	
SD	3 (9.7%)	3 (9.7%)		5 (16.1%)	7 (22.6%)	
PD	0	2 (6.5%)		2 (6.5%)	7 (22.6%)	
ORR	28 (90.3%)	26 (83.9%)	0.354	24 (77.4%)	16 (51.6%)	0.031
DCR	31 (100%)	29 (93.5%)	0.246	29 (93.5%)	23 (74.2%)	0.040

CR: complete remission; PR: partial remission; SD: stable disease; PD: progressive disease; ORR: objective response rate; DCR: disease control rate.

**Table 3:** Comparison of overall survival rates between the observation group and the control group.

Group	Number of cases	6 months	12 months	24 months
Observation group	31	29 (93.5%)	25 (80.6%)	20 (64.5%)
Control group	31	29 (93.5%)	21 (67.7%)	12 (38.7%)
*P* value		0.694	0.384	0.037

RETRACTED

## Data Availability

The data used to support the findings of this study are available from the corresponding author upon reasonable request.
